The article "Advanced Computing Approach for Modeling and Prediction COVID-19 Pandemic" was retracted in 2023. Reasons: signs of a paper mill; suspected computer-generated content; unreliable results or conclusions; concerns about the data.

# Advanced Computing Approach for Modeling and Prediction COVID-19 Pandemic

**DOI:** 10.1155/2022/6056574

**Published:** 2022-04-14

**Authors:** Sami A. Morsi, Mohammad Eid Alzahrani

**Affiliations:** ^1^Applied College in Abqaiq, King Faisal University, P.O. Box 400, Al-Ahsa 31982, Saudi Arabia; ^2^Al-Neelain University, Sudan; ^3^Faculty of Computer Science and Information Technology, Al Baha University, Saudi Arabia

## Abstract

The emergence of many strains of the coronavirus, including the latest omicron strain, which is spreading at a very high speed, is leading to the World Health Organization's (WHO) concern about the creation of this new mutation. Therefore, there is a strong motivation for modeling and predicting COVID-19 to control the number of cases of the disease. The proposed system for predicting the number of cases of COVID-19 can help governments take precautions to prevent the spread of the disease. In this paper, a statistical logistic growth model was employed to predict the spread of COVID-19 in Australia and Brazil. The datasets were collected from the surveillance systems in Australia and Brazil from March 13, 2020, to December 12, 2021, for 641 days. This proposed method used a tested logistic growth model for the complex spread of COVID-19 and forecasted future values within a time interval of six days. The results of the predicted, cumulative, confirmed cases indicate the robustness and effectiveness of the proposed system, which was categorized by time-dependent dynamics. The coefficient of determination (*R*) metric was used to evaluate the model to predict COVID-19, and the proposed system scored the highest correlation (*R*^2^ = 99%). The proposed system has the potential to contribute to public health by making decisions about how to prevent the spread of COVID-19.

## 1. Introduction

The name COVID-19 was given by the World Health Organization (WHO) for contagious diseases caused by severe acute respiratory syndrome corona virus 2 (SARS-CoV-2). The disease affects people differently, with most cases showing mild symptoms, especially in children and young adults [1, 2]. However, some cases can become severe and dangerous, with about 20% of those infected needing medical care in a hospital. Coronaviruses are a large family of respiratory viruses, and some of these cause fewer diseases than others, such as the common cold, and other more severe diseases, such as Middle East Respiratory Syndrome and severe acute respiratory syndrome. These viruses are easily transmitted to another, unlike other viruses [3].

The availability of effective outbreak prediction models can help to gather crucial information about illnesses that are likely to spread and their possible effects. This gathered data allows governments and other groups to propose strategies to address the hazards posed by pandemics [4]. As a consequence of the COVID-19 pandemic, more than 162 million individuals have been infected, and more than 3.3 million people have died. In comparison to prior outbreaks, COVID-19 has exhibited a nonlinear nature and a variety of characteristics that raise concerns about the efficacy of current conventional models [5].

The article "Advanced Computing Approach for Modeling and Prediction COVID-19 Pandemic" was retracted in 2023. Reasons: signs of a paper mill; suspected computer-generated content; unreliable results or conclusions; concerns about the data.

The forecasting of COVID-19 infection rates has become critical for decision-makers and policymakers all around the world. It is essential to estimate by using established scientific procedures and to calculate the rates as precisely as feasible. A prediction of the number of infections might help policymakers in a variety of ways for a given region to examine its present healthcare capabilities and determine ways to halt and control the spread of COVID-19. Different statistical and machine learning models have been proposed to predict COVID-19 infections and deaths to help health officials make timely decisions. These models have provided better analyses to forecast future COVID-19 cases [6].

Various researchers [7] have conducted numerous studies on epidemic modeling and forecasting to combat this spread and have offered analytical forecasts on the extent and end phase of the spread. Kuniya used the susceptible-exposed-infected-recovered (SEIR) compartmental model to estimate the epidemic peak in order to assess the viability of holding the Summer Olympics in Japan in 2020 [8]. Al-qaness et al. used a modified version of the flower pollination algorithm (FPA), paired with the salp swarm algorithm (SSA), to anticipate the number of confirmed cases of COVID-19 in China for 10 days [9]. Based on heuristics and WHO status reports, Koczkodaj et al. [10] estimated an increase in COVID-19 cases outside China by a particular date to reach 1 million cases. Wu et al. evaluated the scale of the Wuhan epidemic and forecasted the degree of local and worldwide spread [11].

Jelena et al. [12] applied a regression model to predict COVID-19. The datasets were collected from different countries to test the proposed system. Isra et al. [13] proposed exponential smoothing and autoregressive integrated moving average (ARIMA) models to forecast COVID-19. The datasets were collected from Saudi Arabia between March 3, 2020, and April 4, 2021. The prediction errors of the proposed system were very high (root mean square errors of 1,225.9). Nahla et al. [14] used a deep-learning, long short-term memory model (LSTM) and gated recurrent unit (GRU) to forecast COVID-19 in Arab countries, namely, Saudi Arabia, Egypt, and Kuwait, from May 1, 2020, to June 12, 2020. Sina et al. [15] introduced the SEIR model to predict active and fatal cases in the US, China, and Italy over a 30-day period. Gergo et al. [16] developed a smart system-based adaptive network-based fuzzy inference system (ANFIS) to predict COVID-19. The system was designed in Hungary and used over a 90-day period. The statistical models were implemented to predict the number of real-life applications to predict COVID-19 cases based on Johns Hopkins University epidemiological data to forecast COVID-19 [17, 18]. They used ARIMA models to predict infection and recovery cases and presented a hybrid ARIMA model and an *α*-Sutte indicator to predict infection cases in Spain [19, 20]. Other researchers have proposed using ARIMA models to forecast occurrence, death, and recovery rates for 25 different countries [21].

The article "Advanced Computing Approach for Modeling and Prediction COVID-19 Pandemic" was retracted in 2023. Reasons: signs of a paper mill; suspected computer-generated content; unreliable results or conclusions; concerns about the data.

Some researchers have used the applied susceptible-infected-removed (SIR) model [22–25]. Numerous authors have developed functions to predict COVID-19 [26–29] and considered various machine learning algorithms [30–32]. Other used neural network approaches to predict future data [33, 34] and parented Bayesian regression models [35, 36]. Still others used logistic functions to predict COVID-19 [37, 38].

Predicting the long-term impact of COVID-19 is a critical step in predicting its future occurrence. [39] Developing a model for the dissemination and consequences of COVID-19 can be extremely significant in understanding the impact of COVID-19. Its occurrence can be modeled and forecasted using artificial intelligence and classic statistical models [40–43]. A logistic growth model was used in this study's principal to develop an accurate prediction model for cases of COVID-19 in Australia and Brazil that estimates how many confirmed cases and how many deaths would occur in a country over a certain period of time bidirectional long short-term memory (Bi-LSTM). In order to forecast COVID-19, we present an innovative logistic growth model, using the validation approach to test the accuracy of the model for COVID-19 estimation. We tested the resilience of the model's resilience by using COVID-19 datasets from multiple countries.

As the epidemic is progressing, accessible information about COVID-19, including its nature and features, is being gathered. It is well known that the virus tends to modify its nature, creating new variations depending on genetic changes. As a result, further studies are required to identify the most effective measures that can aid in ending the COVID-19 pandemic. The novel contribution of this proposed research is to present an appropriate model for predicting the spread of COVID-19 with accuracy. The system can be used to help WHO monitor COVID-19 or any new generation of diseases.

The article "Advanced Computing Approach for Modeling and Prediction COVID-19 Pandemic" was retracted in 2023. Reasons: signs of a paper mill; suspected computer-generated content; unreliable results or conclusions; concerns about the data.

## 2. Materials and Methods

In this study, the logic function was applied to predict COVID-19. We collected information from WHO data and evaluated the information using time series models. The steps of the proposed model are presented in the following subsections.

### 2.1. Dataset

The datasets were collected from WHO using a web application. We have selected a dataset for two countries (Australia and Brazil) for examining and evaluating the proposed system for predicting cases of infection. The data was extracted from surveillance systems dynamically. The actual datasets used for the model are presented in Table 1.

### 2.2. Proposed Model

The logistic method is a statistical approach commonly applied for predictions in epidemiology. The logistic growth model is approximately exponential smoothing. It is used to reduce the rate of growth for a given output.  Figure 1 shows the logistic functions.

(1) $$\begin{array}{c} \frac{1\;dc}{C\;dt}=r\left(1-\frac{C}{K}\right), \end{array}$$

where*C*: number of active cases of COVID-19*r*: growth rate of active cases of COVID-19*K*: size data of epidemic of COVID-19

(2) $$\begin{array}{c} C=\frac{K}{1+\left(k-c_{0}/c_{0}\right)e^{rt}}. \end{array}$$

This equation is used to find the maximum growth rate of active cases at a particular time

(3) $$\begin{array}{c} t_{p}=\frac{\text{In}\left(k-c_{0}/c_{0}\right)}{r}, \end{array}$$

(4) $$\begin{array}{c} C_{p}=\frac{K}{2}. \end{array}$$

Equation (4) is applied to find peak active cases, and the growth rate for analyzing the maximum peak is defined in

(5) $$\begin{array}{c} \frac{dc}{{dt}_{p}}=\frac{rk}{4},\\ c=\frac{b_{1}}{1+b_{2^{e-bZt}}}, \end{array}$$

where *b*_*t*_ is the prediction value from the observation data.

## 3. Experiment Results

In this section, we present the prediction results of the logistic function. The dataset was gathered dynamically during the application. We have taken datasets for two countries (Australia and Brazil). Our objective was to forecast the future value of COVID-19 cases for these countries, and we determined that the actual and predicted values were very close.

### 3.1. Model Evaluation Criteria

The performance measurements, namely, *R*-squared and root mean square error (MSE), were used for the prediction analysis.

(6) $$\begin{array}{c} RMSE=\sqrt{\frac{1}{N}\overset{n}{\underset{i=1}{\sum }}{\left(x_{i}-{\bar{x}}_{i}\right)}^{2}},\\ R^{2}=1-\frac{\sum {\left(x_{i}-{\bar{x}}_{i}\right)}^{2}}{\sum {\left(x_{i}-{\bar{x}}_{i}\right)}^{2}\;}\times 100\%, \end{array}$$

where*x*_*t*_:observation data or actual cases${\bar{x}}_{t}:$predict data*N*: number of sample

The article "Advanced Computing Approach for Modeling and Prediction COVID-19 Pandemic" was retracted in 2023. Reasons: signs of a paper mill; suspected computer-generated content; unreliable results or conclusions; concerns about the data.

### 3.2. Statistical Analysis

A logistic regression model was applied to track the confirmed cumulative cases in Australia and Brazil. The system dynamic is from the WHO website. The simulation estimated the data required to predict COVID-19 cases.  Table 2 shows the estimated coefficients of the proposed system to predict COVID-19 cases in Australia and Brazil.

Initial guess values are *K* = 237303, *r* = 0.0173805, and *A* = 1952.11; the estimation error of the proposed system to predict confirmed cases in Australia is presented. The sum of squares for the residual of the proposed system are 3.9706e -16, 1.706e -05, and 1.1598e -13.

Table 3 summarizes the statistical analysis of the proposed system to predict active cases in Brazil. The initial guess values of the parameters are *K* = 2.21772e + 07, *r* = 0.0394031, and *A* = 479998. The estimation errors were less (*r* parameter = 0.0099521), and the sum square for residual errors was even less (*r* parameters = 4.9348e − 05).

### 3.3. Prediction Results

The logistic regression model was examined to predict confirmed cases of COVID-19 in Australia and Brazil from March 13, 2021, to December 12, 2021. This research will examine the COVID-19 pandemic in Australia and Brazil using the data from the WHO's real reports of infected cases from the earliest confirmed cases to the end of December 2020. Three parameters (*C*, *r*, and *K*) are estimated using a nonlinear, least-squares method. The researchers also examined epidemic “turning points,” the points at which the growth rate of infected people changes from increasing to declining. The study will look at countries that have passed (or are about to pass) epidemic turning points (or epidemic peak points) on the S-curve, are in the middle of an epidemic (or will be in the middle of an epidemic), or have not yet passed (or are still in the epidemic phase). A good fit between the predicted findings and actual data is likely to occur due to the fact that there are countries that are in the late stages of an epidemic based on these features; hence, all parameters of the model are provided.

Table 4 shows the estimation parameters of the logistic function used to predict COVID-19. The prediction tuning time of the COVID-19 pandemic in Australia began in June 2020, whereas it began in July 2020 in Brazil. This indicates that it had approximately 22,177,059 and 227,382 confirmed cases in Australia and Brazil, respectively. The prediction results of the proposed system are very close to the observation data. The estimated peak ratios of confirmed cases obtained by the proposed system are 60,475 for Australia and 8,983 for Brazil.

The article "Advanced Computing Approach for Modeling and Prediction COVID-19 Pandemic" was retracted in 2023. Reasons: signs of a paper mill; suspected computer-generated content; unreliable results or conclusions; concerns about the data.

Table 5 shows the simulation results of the proposed system. It is noted that there is a strong relationship between the actual data and prediction; the percentage of *R*-squared to prediction values in Australia was *R*^2^ = 88.9% and for Brazil was *R*^2^ = 99%.

Figure 2 shows the logistic growth model used to predict confirmed cases in Australia compared with the actual data. The prediction curve shows the total infections of 230,768 and total deaths of 20,106 until December 21, 2021. The graph shows that the cumulative cases will decrease in the upcoming days. The prediction curve has two lines, red and black; these lines represent the prediction errors, whereas the green lines show the size of the infection data at the last stages of COVID-19. The red lines in the middle intersect with confirmed cases to predict the peak unit of COVID-19. The *x*-axis represents the dates, and the *y*-axis represents the number of infections.

The logistic growth model to predict COVID-19 in Brazil is presented in Figure 3. The graphic representation has shown the prediction results of the proposed system to predict cumulative cases in Brazil. The red and black lines represent the prediction output errors. The size of confirmed cases is shown in the green line. The peak point of the epidemic is the intersection close to 02/13/202.

### 3.4. Short-Term Forecasting

In this section, to validate the logistic model, we have forecasted future confirmed cases of COVID-19. The duration for forecasting future cases was from December 7, 2021, to December 18, 2021, in Australia.  Table 6 shows the forecasting values of cumulative cases in Australia. At the beginning, we forecasted future values of confirmed cases from December 7, 2021, to December 12, 2021, and we present actual values for the testing model. We observed that forecasting errors were much less. Subsequently, we applied the logistic model to forecast unseen cumulative COVID-19 cases.

The forecasted, cumulative, confirmed cases of COVID-19 in Brazil are presented in Table 7. We have validated the proposed from December 7, 2021, to December 18, 2021. The forecasting results demonstrated that the forecasting results were very close to the actual values. The performance of the proposed system has indicated the effectiveness of the proposed system in predicting the confirmed and death cases for any country. Finally, we believe the logistic model for predicting COVID-19.

According to the logistic growth model, the correlation coefficient was used to forecast the number of active cases presented in Figure 4. As can be seen, the regression plot closely approximates the actual and test values. Correlation coefficient metrics show that all countries have high correlation coefficient values. This shows that the logistic growth model has a strong relationship with the observed data. There was a 99.39% correlation between the real data and the predicted data in this case. These plots were used to determine the Pearson's correlation between predicted and observed values. Target values are represented by *x*-axis values, whereas output (*y*-axis) values are represented by forecast values.

The article "Advanced Computing Approach for Modeling and Prediction COVID-19 Pandemic" was retracted in 2023. Reasons: signs of a paper mill; suspected computer-generated content; unreliable results or conclusions; concerns about the data.

## 4. Conclusion

The goal of the proposed research is to explore and measure the usefulness of national governments' preventive measures to control the spread of COVID-19, while the new corona mutant reappears on the scene and raises new fears, with a rise in deaths. Therefore, modeling and forecasting the COVID-19 and types of COVID-19 can help WHO limit the spread of this disease. Short-term forecasts of the spread of COVID-19 in Australia and Brazil were demonstrated using a stochastic approach. The prediction of confirmed cases lasted from March 13, 2020, to December 12, 2021, for 641 days. The proposed system used predictions based on cumulative confirmed cases for these countries.

The results show a significant value for measuring and predicting COVID-19 efficiently. In this study, we forecasted the future values for six days, from December 13, 2021, to December 18, 2021, for examining the proposed model. In the training process, there were fewer prediction errors, which proved the robustness of the proposed system to predict COVID-19. Finally, the study confirmed the dynamic use for future preparations of WHO to use the mathematical prediction models to predict the number of confirmed cases for informing counties to find solutions and limit the spread of any disease that appears in the world. Furthermore, the logistic growth model has shown high-performance results to predict COVID-19-confirmed cases and deaths. This model can be very useful for forecasting future data for any disease.

## Figures and Tables

**Figure 1:** Logistic function: (a) exponential growth and (b) logistic growth.

**Figure 2:** Performance of proposed system in Australia: (a) prediction plot and (b) histogram error.

**Figure 3:** Performance of proposed system in Brazil: (a) prediction plot and (b) histogram error.

**Figure 4:** Regression plot of logistic growth model for predicting COVID-19 cases in (a) Australia and (b) Brazil.

**Table 1:** Datasets.

Country	Start date	End date	Number of cases	Number of deaths
*Australia*	03/13/2020	12/12/2021	230,768	2,106
*Brazil*	03/31/2020	12/12/2021	22,177,059	616,457

**Table 2:** Statistical analysis of the proposed system for Australia.

Parameters	Estimated	SE	Tsate	*P*-value
*K*	7.2196e+07	3.9706e -16	1.8183e+23	0
*R*	0.010474	1.706e -05	613.93	0
*A*	2.4664e+05	1.1598e -13	2.1266e+18	0

The article "Advanced Computing Approach for Modeling and Prediction COVID-19 Pandemic" was retracted in 2023. Reasons: signs of a paper mill; suspected computer-generated content; unreliable results or conclusions; concerns about the data.

**Table 3:** Statistical analysis of the proposed system for Brazil.

Parameters	Estimated	SE	Tsate	*P*-value
*k*	2.4281e+07	3.4017e -06	7.138e+12	0
*r*	0.0099635	4.9416e -05	1 201.63	0
*A*	39.262	0.7392	53.115	1.4446e -236

**Table 4:** Significant parameters of the logistic model to predict COVID-19.

Parameters	Australia	Brazil
Number of confirmed cases	22,177,059	227,382
Number of deaths cases	616,457	2,100
Estimated epidemic size	24,306,885	3,408,622
Estimated initial state	604,621	294
Estimated initial doubling time (day)	604,621	65.8
Estimated duration of fast growth phase	69.6	379
Estimated peak date	368	887
Estimated peak rate	60,475	8,983
Estimated end of transition phase	736	1,774

**Table 5:** Estimated results of the logistic model to predict COVID-19.

Number of observation days	Countries	RMSE	*R* ^2^%	F-statistic vs. zero model
641	Australia	*1.68*	*89.4*	*9.36*
641	Brazil	*5.25e+05*	*99.6*	*1.96e+05*

**Table 6:** Short-term forecasting—proposed system in Australia.

Date	Actual	Predicted	Errors
12/07/2021	*222,260*	*224,338*	*0.93*
12/8/2021	*223,914*	*226,599*	*1.20*
12/09/2021	*225,625*	*228,880*	*0.44*
12/10/2021	*227,382*	*231,183*	*0.67*
12/11/2021	*228,925*	*233,506*	*2.00*
12/12/2021	*230,768*	*235,850*	*2.20*
12/13/2021		*230,973*	
12/14/2021		*240,602*	
12/15/2021		*243,010*	
12/16/2021		*245,440*	
12/17/2021		*247,891*	
12/18/2021		*250,365*	

**Table 7:** Short-term forecasting—proposed system in Brazil.

Date	Actual	Predict	Errors
07-Dec-2021	*22,157,726*	*22,449,934*	*1.32*
08-Dec-2021	*22,167,781*	*22,463,372*	*1.33*
09-Dec-2021	*22,177,059*	*22,476,689*	*1.35*
10-Dec-2021	*22,177,059*	*22,489,887*	*1.41*
11-Dec-2021	*22,177,059*	*22,502,966*	*1.47*
12-Dec-2021	*22,177,059*	*22,515,927*	*1.53*
13-Dec-2021		*22,528,771*	
14-Dec-2021		*22,541,499*	
15-Dec-2021		*22,554,112*	
16-Dec-2021		*22,566,610*	
17-Dec-2021		*22,578,996*	
18-Dec-2021		*22,591,269*	

## Data Availability

The datasets were collected from WHO site by using web application. We have selected dataset from two countries, namely, Australia and Brazil, for examining and evaluating the proposed system for predicting infection cases. The dataset is variable in public repository https://www.kaggle.com/imdevskp/corona-virus-report.

## References

[1] Yang P., Liu P., Li D., Zhao D. (2020). Corona virus disease 2019, a growing threat to children?. *The Journal of Infection*.

[2] Watson G. L., Xiong D., Zhang L. (2021). Pandemic velocity: forecasting covid-19 in the us with a machine learning and Bayesian time series compartmental model. *PLoS Computational Biology*.

The article "Advanced Computing Approach for Modeling and Prediction COVID-19 Pandemic" was retracted in 2023. Reasons: signs of a paper mill; suspected computer-generated content; unreliable results or conclusions; concerns about the data.

[3] Theyazn H., Aldhyani H., Joshi M. R., AlMaaytah S. A., Alqarni A. A., Alsharif N. (2021). Using sequence mining to predict complex systems: a case study in influenza epidemics. *Complexity*.

[4] Aldhyani T. H., Alrasheed M., Alqarni A. A., Alzahrani M. Y., Alahmadi A. H. (2021). Deep learning and holt-trend algorithms for predicting covid-19 pandemic. *Computers, Materials & Continua*.

[5] Kermack W. O., McKendrick A. G. (1927). Contributions to the mathematical theory of epidemics. *Proceedings of the Royal Society of London. Series A, Containing Papers of a Mathematical and Physical Character*.

[6] Aldhyani T. H. H., Alkahtani H. (2021). A bidirectional long short-term memory model algorithm for predicting COVID-19 in gulf countries. *Life*.

[7] Boccaletti S., Ditto W., Mindlin G., Atangana A. (2020). Modeling and forecasting of epidemic spreading: the case of COVID-19 and beyond. *Chaos, Solitons and Fractals*.

[8] Kuniya T. (2020). Prediction of the epidemic peak of coronavirus disease in Japan, 2020. *Journal of Clinical Medicine*.

[9] Al-qaness M. A., Ewees A. A., Fan H., Abd El Aziz M. (2020). Optimization method for forecasting confirmed cases of COVID-19 in China. *Journal of Clinical Medicine*.

[10] Koczkodaj W. W., Mansournia M. A., Pedrycz W. (2020). 1,000,000 cases of COVID-19 outside of China: the date predicted by a simple heuristic. *Global Epidemiology*.

[11] Wu J. T., Leung K., Leung G. M. Nowcasting and forecasting the potential domestic and international spread of the 2019-nCoV outbreak originating in Wuhan, China: a modelling study.

[12] Musulin J., Baressi Šegota S., Štifanić D. (2021). Application of artificial intelligence-based regression methods in the problem of COVID-19 spread prediction: a systematic review. *International Journal of Environmental Research and Public Health*.

[13] Al-Turaiki I., Almutlaq F., Alrasheed H., Alballa N. (2021). Empirical evaluation of alternative time-series models for COVID-19 forecasting in Saudi Arabia. *International Journal of Environmental Research and Public Health*.

[14] Omran N. F., Abd-el Ghany S. F., Saleh H., Ali A. A., Gumaei A., Al-Rakhami M. (2021). Applying deep learning methods on time-series data for forecasting COVID-19 in Egypt, Kuwait, and Saudi Arabia. *Complexity*.

[15] Ardabili S. F., Mosavi A., Ghamisi P. (2020). COVID-19 outbreak prediction with machine learning. *Algorithms*.

[16] Pinter G., Felde I., Mosavi A., Ghamisi P., Gloaguen R. (2020). COVID-19 pandemic prediction for Hungary; a hybrid machine learning approach. *Mathematics*.

[17] Box G. E., Jenkins G. M., Reinsel G. C., Ljung G. M. (2015). *Time Series Analysis: Forecasting and Control*.

The article "Advanced Computing Approach for Modeling and Prediction COVID-19 Pandemic" was retracted in 2023. Reasons: signs of a paper mill; suspected computer-generated content; unreliable results or conclusions; concerns about the data.

[18] Ceylan Z. (2020). Estimation of COVID-19 prevalence in Italy, Spain, and France. *Sci Total Environ*.

[19] Chintalapudi N., Battineni G., Amenta F. (2020). COVID-19 virus outbreak forecasting of registered and recovered cases after sixty day lockdown in Italy: a data driven model approach. *Journal of Microbiology, Immunology, and Infection*.

[20] Yue X.-G., Shao X.-F., Li R. Y. M. (2020). Risk prediction and assessment: duration, infections, and death toll of the COVID-19 and its impact on China’s economy. *Journal of Risk and Financial Management*.

[21] Ankarali H., Erarslan N., Pasin O. (2020). Modeling and short-term forecasts of indicators for COVID-19 outbreak in 25 countries at the end of march. *Bangladesh Journal of Medical Science*.

[22] Kermack W. O., McKendrick A. G. (1991). Contributions to the mathematical theory of epidemics—I. 1927. *Bulletin of Mathematical Biology*.

[23] Kermack W. O., McKendrick A. G. (1991). Contributions to the mathematical theory of epidemics—II. The problem of endemicity. 1932. *Bulletin of Mathematical Biology*.

[24] Kermack W. O., McKendrick A. G. (1991). Contributions to the mathematical theory of epidemics—III. Further studies of the problem of endemicity. 1933. *Bulletin of Mathematical Biology*.

[25] Enserink M., Kupferschmidt K. (2020). With COVID-19, modeling takes on life and death importance. *Science*.

[26] Li L., Yang Z., Dang Z. (2020). Propagation analysis and prediction of the COVID-19. *Infectious Disease Modelling*.

[27] Ciufolini I., Paolozzi A. (2020). Mathematical prediction of the time evolution of the COVID-19 pandemic in Italy by a Gauss error function and Monte Carlo simulations. *The European Physical Journal Plus*.

[28] Pham H. (2020). On estimating the number of deaths related to Covid-19. *Physics*.

[29] Cakir Z., Savas H. B. (2020). A mathematical modelling approach in the spread of the novel 2019 Coronavirus SARS-CoV-2 (COVID-19) pandemic. *Electronic Journal of General Medicine*.

[30] Alimadadi A., Aryal S., Manandhar I., Munroe P. B., Joe B., Cheng X. (2020). Artificial intelligence and machine learning to fight COVID-19. *Physiological Genomics*.

[31] Tarnok A. (2020). Machine learning, COVID-19 (2019-nCoV), and multi-OMICS. *Cytometry*.

[32] Wynants L., Van Calster B., Collins G. S. (2020). Prediction models for diagnosis and prognosis of covid-19 infection: systematic review and critical appraisal. *British Medical Journal*.

[33] Singh D., Kumar V., Kaur M. (2020). Classification of COVID-19 patients from chest CT images using multi-objective differential evolution-based convolutional neural networks. *European Journal of Clinical Microbiology & Infectious Diseases*.

The article "Advanced Computing Approach for Modeling and Prediction COVID-19 Pandemic" was retracted in 2023. Reasons: signs of a paper mill; suspected computer-generated content; unreliable results or conclusions; concerns about the data.

[34] Naude W. (2020). Artificial intelligence vs COVID-19: limitations, constraints and pitfalls. *AI & Society*.

[35] National Center for Immunization and Respiratory Diseases (NCIRD) Covid-19 Forecasts. https://www.cdc.gov/coronavirus/2019-ncov/covid-data/forecasting-us.html.

[36] Sperrin M., Grant S. W., Peek N. (2020). Prediction models for diagnosis and prognosis in Covid-19. *British Medical Journal*.

[37] Umaña-Hermosilla B., de la Fuente-Mella H., Elórtegui-Gómez C., Fonseca-Fuentes M. (2020). Multinomial logistic regression to estimate and predict the perceptions of individuals and companies in the face of the COVID-19 pandemic in the Ñuble region, Chile. *Sustainability*.

[38] Ding C., Liu W. (2021). Analysis and prediction for confirmed COVID-19 cases in Czech Republic with uncertain logistic growth model. *Symmetry*.

[39] Cook S., Conrad C., Fowlkes A., Mohebbi M. (2011). Assessing Google flu trends performance in the United States during the 2009 influenza virus A (H1N1) pandemic. *PLoS One*.

[40] Vynnycky E., White R. (2010). *An Introduction to Infectious Disease Modelling*.

[41] Alsaade F. W., Aldhyani T. H. H., Al-Adhaileh M. H. (2021). Developing a recognition system for classifying covid-19 using a convolutional neural network algorithm. *Computers, Materials & Continua*.

[42] Rustam F., Reshi A. A., Mehmood A. (2020). COVID-19 future forecasting using supervised machine learning models. *IEEE Access*.

[43] Ochodek M., Kopczyńska S., Staron M. (2020). Deep learning model for end-to-end approximation of COSMIC functional size based on use-case names. *Information and Software Technology*.

